The article "Fusion of EEG-Based Activation, Spatial, and Connection Patterns for Fear Emotion Recognition" was published in 2022. Journal: Comput Intell Neurosci.

# Fusion of EEG-Based Activation, Spatial, and Connection Patterns for Fear Emotion Recognition

**DOI:** 10.1155/2022/3854513

**Published:** 2022-04-13

**Authors:** Jiahui Pan, Fuzhou Yang, Lina Qiu, Haiyun Huang

**Affiliations:** ^1^School of Software, South China Normal University, Guangzhou 510641, China; ^2^Pazhou Lab, Guangzhou 510330, China

## Abstract

At present, emotion recognition based on electroencephalograms (EEGs) has attracted much more attention. Current studies of affective brain-computer interfaces (BCIs) focus on the recognition of happiness and sadness using brain activation patterns. Fear recognition involving brain activities in different spatial distributions and different brain functional networks has been scarcely investigated. In this study, we propose a multifeature fusion method combining energy activation, spatial distribution, and brain functional connection network (BFCN) features for fear emotion recognition. The affective brain pattern was identified by not only the power activation features of differential entropy (DE) but also the spatial distribution features of the common spatial pattern (CSP) and the EEG phase synchronization features of phase lock value (PLV). A total of 15 healthy subjects took part in the experiment, and the average accuracy rate was 85.00% ± 8.13%. The experimental results showed that the fear emotions of subjects were fully stimulated and effectively identified. The proposed fusion method on fear recognition was thus validated and is of great significance to the development of effective emotional BCI systems.

## 1. Introduction

Emotion is a person's internal reaction to the external environment and plays a crucial role in his or her daily life [1]. Affective computing attempts to endow computers with the capacity to recognize, understand, and express human emotions [2]. At present, there have been certain research results on emotion recognition using physical signals (e.g., facial expressions and verbal speech) and biological signals (e.g., electroencephalogram (EEG)) [3–5]. Compared with nonphysiological signals, EEG signals provide a more objective understanding of emotional processes and responses [6].

In recent years, EEG-based emotion detection has attracted increasing research interest. In these studies [7, 8], EEG-based emotion recognition mainly detected happy and sad emotions, and few studies have directly aimed at the detection of fear emotions. de Man and Stassen [9] analyzed the psychological and physiological responses of fear stimuli using one single-sensor EEG, and the results showed a significant difference between the number of brainwave peaks in a calm state and a fearful state (*p* < 0.05). Masood and Farooq [10] proposed a method for analyzing fear emotion brain signals based on common spatial pattern (CSP) and linear discriminant analysis (LDA) and achieved an accuracy of 74.81% in eight channels and 76.81% in fourteen channels.

Due to the complexity of emotions, EEG-based affective computing relies on the exact EEG features associated with emotions. Researchers have focused on finding the key channels and their interrelationships for EEG-based emotion recognition using different methods. When subjects are undergoing a transition in their emotional state, certain energy differences in the activation patterns of various regions of the brain are detected. Bong et al. [11] analyzed the six emotional states of stroke patients, extracted activation features of five frequency bands by using the wavelet packet transform technique, and achieved a classification accuracy of 82.32% in the beta band. Zheng et al. [12] distinguished different emotional states using differential entropy (DE) and found that the lateral temporal areas had more activities in the beta and gamma bands for positive emotions than those in negative emotions. It should be noted that all the mentioned studies were only based on the analysis of neural activation patterns.

In fact, current studies [13, 14] have revealed that spatial distribution and functional connection features are also important in emotion recognition. On the one hand, the brain function network connection pattern can reflect the connection of various brain areas when transmitting information in emotion recognition [15]. The network function connection is usually used to describe the mechanism of brain network activity. It can be studied by analyzing the time series of EEG data to obtain synchronization between EEG signals. Dasdemir et al. [16] used the phase lock value to detect the brain function connection pattern of conquering emotions. Their results showed that the phase synchronization value between the positive, negative, and neutral emotional channels was significant. The study of emotion recognition based on the functional connectivity pattern of EEG signals can help people understand the potential neural mechanism of emotion processing in the brain.

On the other hand, the spatial distribution model is suitable for EEG emotional classification, and the spatial distribution features can provide more relevant emotional information for identifying different emotional states [17]. CSP is a commonly used strong spatial filtering method that can effectively construct an optimal spatial filter to distinguish two types of EEG data and can effectively extract the eigenvalues of the two types of spatial patterns. Yan et al. [18] proposed an improved CSP method for EEG emotion recognition and achieved average accuracy rates of 85.85% and 94.13%, respectively. Hatamikia and Nasrabadi [19] proposed a simple EEG-based emotion recognition system based on two different public space mode channel reduction methods. Their experimental results show that the spatial pattern algorithm can effectively extract spatially distributed component information from multichannel EEG signals, and the accuracy of distinguishing between fear and neutral emotion reaches 81.48%.

Taken together, EEG-based activation, spatial and connection patterns obtain complementary information on EEG signals during emotional transformation from various aspects. In this study, we propose a fear emotion recognition system based on the fusion of the three EEG-based patterns. Specifically, the DE feature of the activation pattern, the CSP feature of the spatial pattern, and the PLV feature of the connection pattern are extracted and combined. Fifteen healthy subjects joined our experiment and had an average accuracy of 85.00% ± 8.13%, indicating that the emotions of the subjects were fully induced and effectively recognized.

The paper is organized in the following manner.  Section 2 introduces the methods, including subjects, the data acquisition procedure, stimulus materials, graphical interface, experimental paradigm, data processing, and algorithm. The experiments and results are described in Section 3. The discussion and conclusion are presented in Section 4 and Section 5, respectively.

## 2. Method

### 2.1. Subjects

Fifteen healthy subjects (H1 to H15, age 21–37 years, mean age 26 ± 3.8 years, 7 females) from South China Normal University took part in this study after providing written informed consent. All healthy subjects must not only have a normal or corrected-to-normal vision but also have normal hearing.

### 2.2. Data Acquisition

In this study, EEG signals were collected by using the Synamps2 amplifier of the ESI NeuroScan System (Compumedics, Neuroscan, Inc., Australia). Subjects wore a 32-channel EEG cap, and the electrode position conformed to the international 10–20 system placement. However, in this study, we recorded EEG signals in 30 channels. Twelve symmetric electrodes (Fp1-Fp2, F7–F8, F3–F4, FT7-FT8, FC3-FC4, T7-T8, P7–P8, C3–C4, TP7-TP8, CP3-CP4, P3–P4, and O1–O2) and 6 central axis electrodes (Fz, FCz, Cz, CPz, Pz, and Oz) were used. This electrode configuration only excluded reference electrodes A1 and A2. Using the right mastoid as a reference, the ground electrode was placed on the subjects' foreheads. The EEG signal was amplified and sampled at a frequency of 250 Hz. During data acquisition, the impedance of all electrodes was kept below 5 kΩ.

### 2.3. Stimulus Materials

In this experiment, we chose horror movie clips and neutral videos as stimulus videos to quickly and effectively evoke the subjects to produce specific emotional states (fear and neutral, respectively). Fear video clips were mainly from famous fear movies from various countries, including “The Grudge,” “The Conjuring 2,” “Bunshinsaba,” “The Bride,” “The Haunted Apartments,” “It: Chapter One,” “MaMa,” “Terrified,” etc. Neutral videos are mainly from “World Heritage in China Documentary.” The selection process of the video clips was as follows: first, we collected 100 video clips containing horror or neutral scenes from horror movies or short films at home and abroad. Next, the duration of each segment was clipped to approximately 30 seconds, and the total power value was adjusted to match the audio power level of all segments. Then, 10 volunteers (not joined in the BCI experiment) were recruited and asked to evaluate their emotions and indicated a level (no, slight, or extreme) and a keyword (fear or neutral) to describe their emotions while watching the video. Ultimately, the volunteers selected 40 video clips that were considered extremely scary or clearly neutral. Each emotion sort (fear and neutral) included 20 segments.

### 2.4. Graphical Interface and Experimental Paradigm

The experiment was carried out in a dimly lit laboratory. Before starting the experiment, each participant was notified of the entire experimental process. Participants were asked to sit on a comfortable chair in front of a 22-inch LED screen. The distance between the display and the participant was approximately 0.5 meters. During the experiment, the participants were asked to watch the video played on the screen attentively and keep it as still as possible. Participants were required to perform 40 trials, in which videos of fearful and neutral emotions were played 20 times each in a random fashion.

Figure 1 shows the experimental paradigm in each trial. At the beginning of each test, an 8-second prompt was presented to each subject. The subject was asked to watch the horror or neutral videos attentively and experience the corresponding emotion. Then, a horror or neutral video was presented for 30 s. The EEG data were collected synchronously. After the video screening, feedback on a fearful or calm cartoon face based on the online classification was displayed on the screen. The feedback time was 5 seconds, and the rest time was 10 seconds.

### 2.5. Data Processing and Algorithm

In this study, the data processing is shown in Figure 2. Specifically, the EEG data were copied and then fed into three feature selection procedures simultaneously. The analysis methods and algorithms used in this study are described in the following.

#### 2.5.1. Preprocessing

The raw EEG data collected in the experiment were usually accompanied by artifacts, such as electrooculography (EOG) and electromyography (EMG). The data baseline was first corrected by subtracting the mean value of the 1 s signal before the stimulus started. To reduce noise, we then applied a notch filter to remove the 50 Hz power-line noise. Next, a tenth-order bandpass filter between 0.1 and 70 Hz was used in this study.

#### 2.5.2. Feature Extraction

Based on the filtered data, we first calculate the power density spectrum of each channel using a discrete Fourier transform. During the Fourier analysis, we used the zero-padding method to increase the number of data points to 1024 (a power of 2). Next, the band-power values are computed by averaging values in five frequency bands: delta (1–3 Hz), theta (4–7 Hz), alpha (8–13 Hz), beta (14–30 Hz), and gamma (31–48 Hz).

The original formula of DE is defined as follows:

(1) $$\begin{array}{c} \text{DE}=-\int_{a}^{b}p\left(x\right)\log\left(p\left(x\right)\right)\text{ d}x. \end{array}$$

In this equation, *p*(*x*) represents the probability density function of continuous information, and [*a*, *b*] represents the interval of information value. In this study, we used DE features with a 1-second sliding time window for temporal analysis, and we mainly evaluated the performance of DE features and used classification accuracy as a performance indicator.

The spatial filtering of EEG data is crucial when analyzing brain activity. Spatial filtering is used to enhance task-related neural activities to improve the signal-to-noise ratio of EEG data [20]. In this study, CSP was used to extract spatial features and to distinguish different emotional states caused by the stimulation of fear videos and neutral videos. We copied the EEG data, segmented the EEG data using a 1 s time window, and performed bandpass filtering in five selected frequency bands. Through bandpass filtering, the EEG data fragments of each channel and each frequency band are extracted. Then, each EEG data segment undergoes CSP transformation, and the obtained features are used for classification. First, we need to use the two types of emotions corresponding to fear and neutral emotional states in the training data to obtain the CSP spatial filter F. Then, we use this filter to extract the CSP features of each trial:

(2) $$\begin{array}{c} \text{fv}=\;\log_{10}\left(\text{diag}\left(\bar{F}\;{\text{EE}}^{T}{\bar{F}}^{T}\right)\right), \end{array}$$

where fv is the feature vector, $\bar{F}$ is the submatrix formed by selecting the first three rows and the last three rows of *F*, and $\text{diag}\left(\bar{F}\;{\text{EE}}^{T}{\bar{F}}^{T}\right)$ is the EEG data matrix corresponding to one experiment. In formula (2), $\bar{F}\;{\text{EE}}^{T}{\bar{F}}^{T}$ is the vector consisting of all items on the diagonal of matrix *E*, and the logarithm of each item in the vector is calculated by the operator log_10_(.). In this study, to better distinguish the categories of fear and neutral emotional states, we selected the first three components and the last three components from *F*. In addition, by calculating their logarithmic variance, a 6-dimensional feature vector of each frequency band was constructed. Then, the CSP feature vectors of all frequency bands are concatenated to obtain the feature vector of an experiment.

In this study, the phase lock value (PLV) is used to address the synchronization problem of the nonlinear phase. We select the sliding time window with a step of 0.4 s to calculate the PLV. Assuming that the instantaneous phases of the two signals *x*(*t*) and *y*(*t*) are *ϕ*(*x*) and *ϕ*(*y*), the PLV is defined as follows:

(3) $$\begin{array}{c} \text{PLV}=\frac{1}{N}\left|\sum_{j=1}^{N}e^{i\Delta \phi \left(t\right)}\right|, \end{array}$$

where *j* indexes the trial number, *N* is the total number of trials in the process and Δ*ϕ*(*t*) is defined as follows:

(4) $$\begin{array}{c} \Delta \phi \left(t\right)=\phi_{x}\left(j\Delta t\right)-\phi_{y}\left(j\Delta t\right), \end{array}$$

and represents the instantaneous phase difference between the signals *x*(*t*) and *y*(*t*). *ϕ*_*x*_(*j*Δ*t*) and *ϕ*_*y*_(*j*Δ*t*) are the instantaneous phases of the signals in *x* and *y*, respectively. Δ*t* is the sampling period, and *j* is the *j*th sample point. Through (3), the average PLV of all tests can be calculated. When the value of PLV is zero, the phases of the two signals are not coupled, and a PLV of 1 means that the signals are fully coupled. Based on the calculation of the PLV of the brain function connection network, we proposed an EEG-based network pattern (ENP) feature based on EEG data. When estimating the ENP feature, we used the same frequency band and time window to extract the DE feature and CSP feature. In this study, we defined the extracted ENP, DE, and CSP features to utilize their complementary information.

#### 2.5.3. Classification

In this study, we inputted the extracted features into the SVM classifier. During training, all *n* EEG signal samples had the same emotional label as the corresponding EEG signal segment. During the test, the predicted emotion label of an EEG signal segment was obtained by calculating the frequency of the predicted label of its corresponding *n* test samples, and the most common emotion prediction label was identified as the prediction of the EEG picture segment label. Finally, the evaluation index indicated the classification accuracy.

## 3. Experiment and Results

To effectively validate our method, we adopted the leave-one-out cross-validation strategy in this experiment. In this strategy, we use all the trials of the same subject as the data set. Each time, only one trial is used as the test set, and the rest are used as the training set; this step is repeated 40 times. Finally, the accuracy rate is calculated by averaging all results.

The classification results of different types of features in the delta, theta, alpha, beta, and gamma bands are shown in Table 1. ENP represents the connection characteristics of brain function, DE describes entropy, CSP describes spatial characteristics, and DE_ENP_CSP is the fusion of the three characteristics. All bands refer to the frequency bands that connect all five frequency bands. The results show that the EEG feature that concatenated DE, CSP, and ENP features in all bands achieve the highest recognition accuracies, except for subjects H3 and H6. In addition, the accuracy of the classifier trained with the DE_ENP_CSP feature is significantly higher than that of the DE, CSP, or ENP feature training alone.

Table 2 shows the average classification accuracy of all healthy subjects. These experiments employed 4 different feature extraction methods. The results showed that the DE feature had a better classification effect in the alpha band. The accuracy of the ENP feature in the beta band was higher than that of the other bands. The effect of the CSP feature in the alpha band was better than that of the other bands, while the accuracy of the DE_ENP_CSP feature in the theta, alpha, and beta bands was better. In addition, for the features based on DE and DE_ENP_CSP, the classification performance of connecting all five-word bands is significantly better than the classification performance of any single frequency band.

Table 3 shows the performance comparison of the single-feature method and the feature-fusion method in each frequency band. The *t* test was used for analysis to determine whether there was a significant difference between the accuracy of feature fusion and the accuracy of a single feature. In all bands, the classification accuracy of the feature fusion method ED_ENP_CSP significantly outperforms the classification accuracy of the single feature method DE, CSP, or ENP, which proves that the performance of the fusion method is better than that of a single feature.

It is difficult to compare the accuracy of obtaining individual emotional states with state-of-the-art because the classes of target emotions identified and the methods used vary between studies.  Table 4 lists the classes of emotion, features, frequency bands, and the corresponding accuracies in the previous studies, which aims to compare the performance of different features in emotion recognition and to explore the frequency bands with more significant activations under different emotional states.

In addition to identifying the classification of emotions, it is also important to understand the brain activation patterns of emotions. We observed the activation state of the brain through a topographic map of the brain. As shown in Figure 3, the classification weight of each electrode was the mean of the weights of all frequency bands. The weight value was determined from the SVM training model. We found that fear emotions were mainly processed in the right hemisphere, showing an asymmetrical phenomenon [27].

To illustrate the neural pattern of fear emotions, we drew a topographic map based on 5 frequency bands.  Figure 4 shows the DE distribution of all subjects, that is, the characteristics of all healthy subjects and the average of all trials. However, the distribution patterns of neural activity activation in different frequency bands between a fearful emotional state and normal emotional state have high similarities. In response to fear emotions, we found that the temporal lobes on both sides were more active in the delta, theta, and alpha bands, and for the gamma band, they were more active in the occipital region. In response to neutral emotions, the right prefrontal region was more active in the five frequency bands.

In addition, we further analyzed the connection mode between different electrodes in different frequency bands. To determine the different connectivity indexes between all 30 electrodes, we used repeated measures analysis of variance (ANOVA) to test whether there were significant differences in the EEG channel connection strength between fear and neutral emotion in different frequency bands.  Figure 5 depicts the associations with significant differences between the fear and neutral emotional states of all subjects. These associations were revealed by a one-way analysis of variance in different frequency bands. In Figure 5, the results show that in the delta and theta bands, there are significantly different connections in the parietal region, while in alpha, there are significantly different connections in the frontal region. In the beta zone, connections with significant differences mainly existed between the nodes in the left temporal lobe, parietal lobe, and occipital lobe. In the gamma zone, it is concentrated between the nodes of the left temporal lobe, parietal lobe, and occipital lobe. There was also little connection between the frontal lobe and the right temporal lobe. Significant differences between the two emotional states mainly appear in the alpha, beta, and gamma bands. These significant differences may further indicate that the features of the alpha, beta and gamma bands have higher classification accuracy.

The CSP spatial filtering method is used to analyze the EEG signals in the spatial domain. We constructed spatial feature vectors of EEG signals under fear and neutral emotions. After CSP spatial filtering, all the EEG data of each participant were visualized, and the EEG signal was drawn with a whole head topographic map, as shown in Figure 6. For the delta band CSP spatial filter, the value of the right frontal lobe region is higher than other frequency bands, while the theta band is significantly different from other frequency bands in the temporal lobe region, and the alpha band has a higher value in the parietal lobe region. The beta band has higher values in the prefrontal lobe and posterior parietal lobe, and the gamma band has higher values in the left frontal region than other frequency bands.

## 4. Discussion

In this study, an EEG-based BCI system for emotion recognition was developed to identify the fear and neutral emotional states of subjects when watching videos. Compared with single-modal features, multimodal features can provide more separable information, which may improve the recognition accuracy [28, 29]. Zheng [12] compared the efficiency of different features in emotion recognition and found that the DE feature achieved the highest classification results. Masood and Farooq [10] proved that CSP features also contain information to distinguish different emotional states. Therefore, in this study, we extracted the single-modal features of DE, CSP, and ENP and further constructed the multimodal features of DE_ENP_CSP. As shown in Table 1, the fusion features of all bands achieved the highest classification accuracies in almost all subjects. This result also shows that the combination of EEG-based activation patterns, spatial patterns, and brain functional connection patterns can improve recognition performance.

Table 2 shows the average recognition accuracies of all 15 healthy subjects in each feature and different frequency bands. The fusion (multimodal) feature of DE_ENP_CSP in all bands achieves the best classification results of 85.00% ± 8.13%. The results in Table 3 show that fear emotion is related to multiband features, and the fusion method performs significantly better than the single feature method (*p* value<0.01). The results in Table 4 show that generally higher frequency bands have better activation emotion results. Meanwhile, from the above comparison with other EEG-based studies, we can infer that our proposed feature extraction method has acceptable classification performance. At the same time, when comparing our results with other EEG-based emotion recognition systems, we found that the same feature method differs in emotion recognition, and different studies have different accuracy ranges. Since we study feature fusion methods based on three different modes, we cannot make precise comparisons with other studies, but it can be found that our fusion feature achieves an average accuracy of approximately 80% in the frequency band, with the most significant activation results, which shows that our fusion method can produce good results.

The high performance of our emotion recognition system may be attributed to the following points. First, since the appropriate stimulus materials play a critical role in inducing emotions, the carefully selected and edited horror movie clips used in this study can more fully simulate participants' fear emotion. Second, the subjects were asked to pay more attention to the task of emotion recognition during the experiment. Finally, we included a period of rest after the end of each video, during which subjects could adopt suitable strategies to adjust their emotions and prepare for the next trial.

Our study also verified proper emotional patterns. As shown in Figure 3, fear emotion was mainly processed in the right hemisphere, which is consistent with the results of previous studies [29, 30]. As presented in Table 2, for the brain activation pattern, the DE feature of the alpha band achieves the highest recognition accuracy rates in all frequency bands. Previous studies have found that subjects have more alpha and beta activations while they are experiencing fear [31]. Regarding the characteristic pattern of brain function connection, when subjects watched tense and panic-inducing movie clips [32], the accuracy of fear emotion recognition in the alpha band was better than that in other bands, which is consistent with the research results of [33]. For the spatial pattern, the recognition accuracy in the alpha band is better than that in the other bands. Notably, when a person experiences fear, his or her muscles will tremble, and electromyography activity is mainly distributed in the high-frequency band [34]. However, through the above analysis, we found that our high recognition accuracy is not caused by myoelectric activity. In conclusion, our emotion recognition BCI system could arouse and identify subjects' fear and neutral emotions well, and that fear emotion has a better classification effect in the alpha band.

The classification results show that the connectivity index of each frequency band contains distinguishable information on fear and neutral emotions. Related research [32] found that the alpha frequency band is associated with emotions, but some studies also found that the frequency band activities of theta [33], beta [34], and gamma [35] are also affected by emotional states. Our results show that functional connections based on EEG signals have a certain correlation with fear emotions in each frequency band. That is, the connection between fear and EEG patterns is not limited to a certain frequency band but has good recognition in all frequency bands. Some related studies also extracted features from all frequency bands to identify the emotional state of the user [36], but these studies did not compare it with the classification performance of extracting features from a single frequency band. The results of Tables 1 and 2 show that features extracted from multiple bands tend to obtain better classification results than single band features. The study by Nie et al. [37] also reached similar results. Moreover, our feature extraction method of fusing three patterns also obtained the best classification effect when connecting five frequency bands. Therefore, for the recognition of fear emotion, it may be better to extract the features from multiple frequency bands rather than just a single frequency band.

As shown in Figure 4, there are certain differences in the activation patterns between fear emotion and neutral emotional states. In general, the degree of activation of fear emotion is higher in the low-frequency band but lower in the high-frequency band than neutral emotion. The activation areas of fear emotion in the delta, theta, and alpha bands are mainly the temporal lobe, parietal lobe, and occipital lobe, while activation areas in the beta and gamma bands are only the parietal and occipital lobes. The neutral emotion had obvious right prefrontal activation in all five frequency bands. The results imply that the activation patterns of different emotional states are different, and there are also certain differences in the activation patterns of the same emotion in different frequency bands.

Brain functional connections represent information transmission among different brain areas. From Figure 5, we can conclude that the connections with significant differences were mainly concentrated in the alpha, beta, and gamma bands. A previous study [38] also showed that negative emotions have a better processing effect in high-frequency bands. In addition, the significantly different connections in the high-frequency range were mainly concentrated in the left temporal lobe, parietal lobe, and occipital lobe. In the low-frequency range, the connection between the parietal lobe and the occipital lobe is stronger. This also shows that in different emotional states, there may be information transmission between different areas of the brain.

It can be seen from the topographic map of the CSP mode in Figure 6 that the spatial distribution of the energy distribution of the fear emotion in different frequency bands is different. The CSP pattern of the delta band is more pronounced on the right unilateral frontal lobe. In the theta band, after processing by the CSP filtering method, the emotional energy is concentrated in the left temporal lobe and posterior occipital lobe. For the alpha band, the emotional energy values are distributed in the frontal lobe, parietal lobe, and occipital lobe. In the beta band, when the CSP spatial filtering method is used, the energy value of emotion is mainly concentrated in the prefrontal lobe. In the gamma band, the energy value of emotion is mainly distributed in the left frontal lobe.

In our daily lives, the emotion of fear is often difficult to judge. We cannot accurately determine whether some of our physiological reactions are caused by fear or other factors. Furthermore, it is difficult to consciously regulate one's emotional state [37]. The ability to self-regulate and calm in a state of fear is conducive to people's physical and mental health. Therefore, the establishment of a BCI detection system for fear emotion can help people better analyze and adjust their emotions.

Although the system has high recognition accuracy in detecting the fear emotions of healthy subjects, it still has certain limitations. First, we only verified our system in a small number of subjects, and their emotions were induced through video. More participants should be recruited, and more emotional stimulus methods should be devised. Second, when extracting features for classification, we only analyzed the classification effects of DE, CSP, ENP, and DE_ENP_CSP and did not analyze the classification performance of other extracted features. Finally, we only used the classification method of SVM, and other classifiers and deep learning methods should be considered. Considering these limitations, we will work to improve our emotional BCI system in the future and develop it into an emotional regulation BCI system.

## 5. Conclusions

In this study, we proposed a method for identifying fear emotions based on EEG data and verified it by using fear videos to induce fear emotions in 15 healthy subjects. The good recognition effect proves the effectiveness of our recognition method. We propose to integrate the functional connection pattern characteristics of the brain network, the activation signs based on EEG signals, and the spatial pattern characteristics to identify fear emotions. We can conclude that the use of EEG signals to establish functional connections between brain regions may be an important way to improve the performance of BCI, reflecting brain emotions in the future.

## Figures and Tables

**Figure 1:** The experimental protocol of our emotion recognition system.

**Figure 2:** Flow chart of emotional recognition. (a) Video-evoked emotional EEG. (b) A feature set was constructed by fusion of DE, CSP, and ENP. (c) Five kinds of frequency features (delta, theta, alpha, beta, and gamma) were selected. (d) Emotion recognition by SVM.

**Figure 3:** Topographical map of the classification weight.

**Figure 4:** Topographical maps of the average DE features of all subjects in the five bands (delta, theta, alpha, beta, and gamma) with fear or neutral emotional states. Note that the top 5 topographic maps are the scalp DE distributions in different frequency bands during the fearful emotional state, and the bottom 5 topographic maps are the scalp DE distributions in different frequency bands during the neutral emotional state.

**Figure 5:** The paired differential networks between fear and neutral emotional states in different frequency bands. Note that the blue line indicates that the synchronization state between the electrodes is significant.

**Figure 6:** Topographic maps of emotions in CSP spatial filtering in different frequency bands.

**Table 1:** Classification accuracy using different features.

Subject	Feature	Delta (1–3 Hz)	Theta (4–7 Hz)	Alpha (8–13 Hz)	Beta (14–30 Hz)	Gamma (31–48 Hz)	All bands
H1	DE	95	92.5	92.5	97.5	97.5	95
	ENP	65	70	95	100	95	85
	CSP	85	97.5	92.5	95	95	97.5
	DE_ENP_CSP	90	97.5	97.5	100	97.5	100

H2	DE	95	95	90	75	75	90
	ENP	75	75	65	75	45	65
	CSP	75	70	85	50	40	80
	DE_ENP_CSP	95	90	85	60	65	92.5

H3	DE	82.5	85	77.5	72.5	87.5	90
	ENP	60	60	64	60	65	57.5
	CSP	90	92.5	95	80	72.5	77.5
	DE_ENP_CSP	85	85	85	77.5	75	87.5

H4	DE	57.5	60	80	75	67.5	85
	ENP	60	60	65	67.5	65	60
	CSP	55	77.5	92.5	72.5	60	90
	DE_ENP_CSP	62.5	85	87.5	80	62.5	92.5

H5	DE	82.5	80	85	82.5	67.5	87.5
	ENP	65	62.5	67.5	65	65	65
	CSP	67.5	65	77.5	72	75	75
	DE_ENP_CSP	72	82.5	87.5	87.5	70	95

H6	DE	70	65	75	65	82.5	82.5
	ENP	65	67.5	67.5	70	70	67.5
	CSP	80	92.5	87.5	70	72	62.5
	DE_ENP_CSP	75	75	75	67.5	75	77.5

H7	DE	62.5	62.5	72.5	75	70	72.5
	ENP	67.5	67.5	67.5	72.5	70	67.5
	CSP	57.5	65	67.5	73.5	70	67.5
	DE_ENP_CSP	67.5	65	70	77.5	72.5	75

H8	DE	62.5	75	80	57.5	67.5	72.5
	ENP	60	60	67.5	67.5	65	60
	CSP	55	73.5	80	75	77.5	82.5
	DE_ENP_CSP	65	70	80	70.75	70	80

H9	DE	67.5	77.5	67.5	47.5	52.5	72.5
	ENP	62	65	65	65	67.5	62.5
	CSP	67.5	40	60	67.5	70	70
	DE_ENP_CSP	65	62.5	67.5	57.5	62.5	75

H10	DE	60	70	70	67.5	65	75
	ENP	60	60	62.5	60	61.75	60
	CSP	70	85	82.5	77.5	75	80
	DE_ENP_CSP	70	77.5	82.5	72.5	75	82.5

H11	DE	75	70	80	82.5	47.5	77.5
	ENP	65	67.5	72.5	72.5	67.5	65
	CSP	57.5	77.5	77.5	77.5	62.5	75
	DE_ENP_CSP	72.5	72.5	80	85	67.5	80

H12	DE	97.5	92.5	92.5	77.5	80	92.5
	ENP	75	75	80	80	75	75
	CSP	67.5	80	80	50	67.5	87.5
	DE_ENP_CSP	87.5	95	90	77.5	75	95

H13	DE	60	60	75	57.5	52.5	72.5
	ENP	70	70	67.5	65	67.5	70
	CSP	70	65	72.5	60	50	70
	DE_ENP_CSP	60	72.5	77.5	65	70	77.5

H14	DE	60	67.5	77.5	62.5	60	77.5
	ENP	60	60	57.5	57.5	55	60
	CSP	57.5	75	67.5	60	42.5	75
	DE_ENP_CSP	57.5	72.5	77.5	57.5	55	82.5

H15	DE	60	70	70	67.5	65	75
	ENP	60	60	62.5	60	61.75	60
	CSP	70	85	82.5	77.5	75	80
	DE_ENP_CSP	70	77.5	82.5	72.5	75	82.5

**Table 2:** The average classification accuracy of different features.

Feature	Delta (0.5–3.5 Hz)	Theta (4–7 Hz)	Alpha (8–13 Hz)	Beta (14–30 Hz)	Gamma (31–48 Hz)	All bands
DE	72.50 ± 14.45	74.83 ± 11.89	79.00 ± 8.01	70.83 ± 12.27	69.17 ± 13.68	81.17 ± 8.18
ENP	64.63 ± 5.27	65.33 ± 5.50	68.43 ± 8.89	69.17 ± 10.59	66.40 ± 10.56	65.33 ± 7.19
CSP	68.33 ± 10.84	76.07 ± 14.37	80.00 ± 10.04	70.53 ± 11.78	66.97 ± 14.26	78.00 ± 9.07
DE_ENP_CSP	72.97 ± 11.43	78.83 ± 10.34	81.67 ± 7.72	73.83 ± 11.73	71.17 ± 9.40	85.00 ± 8.13

**Table 3:** The performance of feature fusion and single-feature extraction.

	Feature	Delta (0.5–3.5 Hz)	Theta (4–7 Hz)	Alpha (8–13 Hz)	Beta (14–30 Hz)	Gamma (31–48 Hz)	All bands
*p* value	DE/DE_ENP_CSP	0.77	0.12	0.07	0.09	0.09	<0.01
	ENP/DE_ENP_CSP	<0.01	<0.01	<0.01	0.09	0.01	<0.01
	CSP/DE_ENP_CSP	0.06	0.41	0.36	0.19	0.09	<0.01

**Table 4:** List of studies using EEG signals to perform emotion recognition.

Studies	Features	Accuracies	Classes of emotion	Relevant frequency bands
Our study	DE	79.00 ± 8.01	Fear	Alpha
			Neutral	Alpha
	CSP	80.00 ± 10.04	Fear/neutral	Alpha
	ENP	69.17 ± 10.59	Fear/neutral	Beta/gamma
	DE_ENP_CSP	81.67 ± 7.72	Fear/neutral	Alpha

Huang et al. [21]	DE	87.00 ± 7.30	Positive	Theta
			Negative	Theta

Pan et al. [22]	CSP	62.92	Happiness/sadness	Gamma

Li et al. [23]	DE	62.37 ± 10.27	Happiness	Beta/gamma
			Disgust	Gamma
			Fear	Alpha
			Sad	Alpha
			Neutral	Alpha

Li et al. [24]	DE	45.10 ± 8.13	Positive	Beta
			Negative	Alpha

Jiang et al. [25]	DE	84.76 ± 14.62	Angry	Theta
			Surprise	Beta/gamma
			Neutral	Theta/alpha

Li et al. [26]	PSD	60.00 ± 0.07	Positive/neutral	Beta
			Negative/neutral	Beta/gamma
	DE	65.00 ± 0.09	Positive/neutral	Beta
			Negative/neutral	Beta/gamma
	ENP	65.00 ± 0.09	Positive/neutral	Beta/gamma
			Negative/neutral	Beta/gamma
	PSD_ENP	68.00 ± 0.07	Positive/neutral/negative	Beta
	DE_ENP	67.00 ± 0.08	Positive/neutral/negative	Gamma

## Data Availability

The data presented in this study are available upon request from the corresponding author.
